# Predicting Divorce Prospect Using Ensemble Learning: Support Vector Machine, Linear Model, and Neural Network

**DOI:** 10.1155/2022/3687598

**Published:** 2022-07-11

**Authors:** Mian Muhammad Sadiq Fareed, Ali Raza, Na Zhao, Aqil Tariq, Faizan Younas, Gulnaz Ahmed, Saleem Ullah, Syeda Fizzah Jillani, Irfan Abbas, Muhammad Aslam

**Affiliations:** ^1^Department of Software Engineering, University of Central, Punjab 54000, 1-Khayaban-e-Jinnah Road, Johar Town, Lahore, Pakistan; ^2^Department of Computer Science, Khwaja Fareed University of Engineering and Information Technology, Rahim Yar Khan 64200, Pakistan; ^3^State Key Laboratory of Resources and Environmental Natural Resources Research, Chinese Academy of Sciences, Beijing 100101, China; ^4^State Key Laboratory of Information Engineering in Surveying Mapping and Remote Sensing, Wuhan University, Wuhan 430079, China; ^5^Department of Physics, Physical Sciences Building, Aberystwyth University, Aberystwyth SY23, UK; ^6^School of Agricultural Equipment Engineering, Jiangsu University, Zhenjiang 212013, China; ^7^School of Computing Engineering and Physical Sciences, University of West of Scotland, Paisley, UK

## Abstract

A divorce is a legal step taken by married people to end their marriage. It occurs after a couple decides to no longer live together as husband and wife. Globally, the divorce rate has more than doubled from 1970 until 2008, with divorces per 1,000 married people rising from 2.6 to 5.5. Divorce occurs at a rate of 16.9 per 1,000 married women. According to the experts, over half of all marriages ends in divorce or separation in the United States. A novel ensemble learning technique based on advanced machine learning algorithms is proposed in this study. The support vector machine (SVM), passive aggressive classifier, and neural network (MLP) are applied in the context of divorce prediction. A question-based dataset is created by the field specialist. The responses to the questions provide important information about whether a marriage is likely to turn into divorce in the future. The cross-validation is applied in 5 folds, and the performance results of the evaluation metrics are examined. The accuracy score is 100%, and Receiver Operating Characteristic (ROC) curve accuracy score, recall score, the precision score, and the F1 accuracy score are close to 97% confidently. Our findings examined the key indicators for divorce and the factors that are most significant when predicting the divorce.

## 1. Introduction

Divorce (or dissolution of marriage) is the definitive termination of a marital partnership, canceling the legal duties and responsibilities of marriage and dissolving the parties' matrimonial relations. In other terms, divorce is a constitutional action taken by married people to end their marriage. It is also known as marriage dissolution and is the constitutional step that ends a marriage ahead when either partner dies.

In general, there are two sorts of divorce. One option is “divorce from bed and board,” which is legal in some jurisdictions. At its essence, this permits couples to legally separate and is frequently utilized by spouses who want to live their own lives but do not want to formally break their marriage for whatever reason. Divorce from bed and board is uncommon these days. An “absolute divorce,” which terminates the marriage, is the most prevalent kind of divorce, therefore, to speak, a legal clean break. This topic will be the subject of this article. There are several ways to achieve the aim of having a court issue, an absolute divorce ruling. For convenience, it has been the usual practice in law to classify each of these procedures as a different type of divorce, which we will do here.

The following states contain divorce data for the United States. There have been 2,015,603 weddings. Marriage occurs at a rate of 6.1 per 1,000 of the population in total. There have been 746,971 divorces. Divorce occurs at a rate of 2.7 per 1,000 people (45 reporting states) [1].

Divorce occurs at a rate of 16.9 per 1,000 married women. Many experts believe that this is a far more authentic representation of the genuine divorce rate [2] than the raw number. The divorce rate for every 1,000 married women is about double of what it was in 1960; nonetheless, it is lower than the all-time high of 22.6 in the early 1980s. In the United States, about half of the total marriages end in separation or divorce. According to the researchers, 41% of all the first marriages result in divorce. The second marriages fail about 60%. All third marriages end in divorce about 73%. The United States has the world's sixth highest divorce rate [3].

Machine learning is an artificial intelligence (AI) technique that enables computers to automatically develop and learn on their own without being explicitly programmed. Machine learning [4] is anxious with the establishment of computer programmers that can access information data and employ it to learn on their own. Text classification [5] is a machine learning approach that assigns tags or categories to text automatically. Text classifiers can evaluate and categorize text by sentiment [6], subject, and consumer intent using natural language processing (NLP) [7] quicker and more correctly than people.

Ensemble modeling is an effective method for improving the performance of our model. It typically pays to use ensemble learning in addition to any other models we may be developing. Ensemble learning techniques [8] are a kind of machine learning methodology that accommodates numerous base techniques to create the best prediction technique.

The divorce prospect prediction is the core objective of this novel research study. The main contributions of this research are the following:

- A novel research study in terms of divorce prospect prediction using a questionnaire dataset is proposed in this paper.
- The three advanced machine learning models, support vector machine (SVM), passive aggressive classifier (PAC), and neural networks (multilayer perceptron classifier) are utilized for the prediction task. Our employed techniques are fully hyperparameter tunned.
- An enhanced novel ensemble learning approach based on three machine learning techniques is employed to predict the divorce prospect of the couple.
- The divorce exploratory data analysis (DEDA) is conducted to get fruitful insights to form the dataset and to determine the major factors that cause divorce.
- The cross-validation (CV) is applied in 5 folds, and the performance results evaluation metric of the proposed approach is examined.
- The comparative analysis of model performance is conducted among the three employed SVM, PAC, and Neural network approaches.

The rest of the paper is formulated as: The divorce-related work is examined in Section 2. The architectural methodology analysis of our proposed research approach is analyzed in Section 3. The applied advanced machine learning techniques are examined in Section 4. Then, a novel ensemble learning approach based on three machine learning techniques is discussed in Section 5. The results and evaluation of the proposed approaches are explained and deliberated in Section 6. Then, to conclude the research work, Section 7 contains the conclusion of this novel research study.

## 2. Related Work

The authors used Yöntem's findings to construct 56 questions as divorce predictors. Furthermore, they employed four automated learning models (perceptron, logistic regression, neural networks, and randomized forest) as well as three hybrid models based on voting criteria. Each of these models was trained in 5 distinct scenarios, resulting in a total of 35 tests, with the performance attained in terms of accuracy, sensitivity, and specificity is 0.98, 1.0, and 0.96, respectively, for the perceptron model and a hybrid model [9].

The categorization approaches are used to forecast divorce in Turkey. In 2019, the authors carried out this investigation. They determined in this study that the ANN technique paired with a correlation-based matrix of feature space selection performs best, with an accuracy score of 98% and a Kappa value of 0.97. The SVM model training span is also less than that of the ANN model training span [10].

The authors utilized significant characteristics in this suggested study by deleting duplicate features that do not help with the prediction by applying an improved machine learning technique to the standard dataset accessible to forecast the divorce rate. They were able to reach 99% accuracy. This technique may also be utilized as evidence by family counseling professionals on a couple's emotional and psychological well-being [11].

Within the area of this study, divorce prediction was performed utilizing the Divorce Predictors Scale based on the Gottman couple's therapy. DPS's success was explored utilizing the multilayer perceptron (MLP) neural networks and decision tree algorithms. The study also seeks to identify the most important features of the Divorce Predictor Scale values that influence divorce. When the direct classification learning methods were applied to the divorce dataset, the RBF neural network had the greatest success rate of 98%. This scale can be used by family counselors and family therapists to help with the case formulation and intervention planning. Furthermore, the predictors of divorce in the Gottman couple relation therapy were verified in the Turkish samples [12].

In a long-term, prospective longitudinal research, this paper explores the predictability of divorce. During the 14-year research period, the prediction was attainable with a technique that incorporated marital happiness, concerns of the marriage breakup, and emotional interaction in both talks. The algorithm correctly predicted divorce 93% of the time [13].

An artificial neural network (ANN) technique was created and employed in this research to predict whether or not a couple will divorce. The prediction is based on several questions that the couple acknowledged, and the answers to those questions served as the input data to the ANN model. The model was subjected to repeated learning over training data and validation cycles until it achieved 100% accuracy [14].

The authors are offering a study on the prediction of divorce cases using available machine learning techniques in this paper. The authors compared the accuracy of the perceptron learning classifier, random forest learning classifier, decision tree learning classifier, Naive Bayes learning classifier, support vector machine learning classifier, and K-nearest neighbor learning classifier for divorce case prediction. Following training, the algorithm will forecast whether or not the divorce will materialize. This allows the therapist to assess how stressful a couple's condition is and properly counsel them. With the perceptron model, the authors attained an accuracy of 98% [15].

The detection of COVID-19 based on a blood test was proposed in this study [16]. The ensemble-learning-based approach was developed for the prediction of COVID-19. At the first stage of research, the deep-learning-based classifier convolutional neural network (CNN) was utilized. The dataset was used from the San Raffaele Hospital. In the second stage of research, the 15 different machine-learning-based classifiers were applied. The findings of the research study show that the ensemble learning model achieved an accuracy score of 99%.

Malware detection based on ensemble learning techniques is proposed in this study [17]. The fully connected convolutional neural network (CNN)-based classifier was developed for base stage classification. The machine-learning-based models were utilized for end-stage classification. 15 machine-learning-based classifiers were utilized for malware detection. The dataset of Windows Portable Executable (PE) malware was used for model training and testing results. The research findings show that the fully connect CNN ensemble model and machine-learning-based extra trees classifier achieved an accuracy score of 100%.

In conclusion, our proposed novel research study is based on the prediction of divorce prospects using ensemble learning techniques. The comparative analysis with the past applied research study shows that our research study outperformed by utilizing advanced techniques. The research study results' outcomes are efficient, validated, and higher than the past applied approaches. We have revealed the key indicators for divorce and the factors that are the most significant when predicting divorce in this research study.

## 3. Methodology

The methodological analysis of the proposed research study is analyzed in this section. The working flow of our research findings flow is elaborated here.

The questionnaire dataset is analyzed and useful insights are taken from it. Feature engineering is applied to make a predictable model with the best-fit features in the context of divorce prediction. The data normalization is applied to make the dataset in perfect form for our proposed model.

Now dataset splitting is applied to split the dataset into two portions. The 80% portion of the data is used for model training and 20% is utilized for model testing and performance evaluation. The three models are applied with the ensemble learning approach. Finally, the ensemble learning model prediction is used for predicting the divorce.

The research methodology for this novel research is examined in Figure 1. It visualizes the workflow of the complete research study. In the first step, the questionnaire dataset is analyzed by the exploratory data analysis (EDA). Then, in the next step, feature engineering is applied to get the useful features for the ensemble learning model. Then, the data normalization is applied. The dataset splitting is applied in the next step. Then, the train portion is given to the model, and then, the test model results in the evaluation of the test portion. After all these methodology steps are done, a predictive ensemble learning model is formed and ready to predict the divorce of a couple.

### 3.1. Dataset

The dataset is based on the questions asked by the specialists to the married couples [18]. The answers to these 54 questions will predict the chance of divorce between them. The questions are graded on a scale of 0 to 4, with 0 being the worst and 4 being the best. The last category indicates whether or not the couple has divorced.  Table 1 contains the descriptive dataset analysis.

### 3.2. Divorce Exploratory Data Analysis

The divorce exploratory data analysis (DEDA) refers to the essential process of administrating preliminary investigations on data to spot anomalies. The uncovered data patterns can be found by applying DEDA. The test hypotheses are performed using DEDA. The assumption validation using graphical representations and summary statistics is demonstrated by utilizing the DEDA.

The bar plot is a plot on the Divorce_Y_N column in Figure 2. In the bar plot, 0 represents the number of divorce class and 1 represents the divorce class. The bar plot shows the total number of divorces and not divorce value. The value of divorce in Figure 2 is 86, and the value of number of divorce is 84. The bar chart shows that the data set is balanced. Both classes have approximately the same number of rows.

The violin chart is the plot based on the dataset to explore the cause of divorce in Figures 3 –5. A violin graph is a cross between a kernel density plot and a box plot that visualizes the data peaks. It is utilized to display how numerical data points are distributed in the employed dataset.

As opposite to a box plot, which can only bring summary statistics, violin graphs visualize summary statistics as well as the frequency of every variable. In the violin plot of the I'm_not_wrong (51) column, we explore that as the intensity of value increases, the number of divorces increases, and as the value decreases, the number of divorces decreases. The analysis graph also shows that it has a great impact on the Divorce_Y_N column.

In Figure 3, the data from the violin plot is also explored with the column of love (16), common goal (10), and enjoy holidays (8). The graph shows the cause of divorce and no_divorce when the value of the scale changes. The violin plot is also plotted on the column of happy (17), always never (32), trust (21), and you are inadequate (53) in Figure 4.

The violin plot shows how the cause of divorce changes when the scale changes. The violin plot of argue_then_leave (42), humiliate (36), and friend social (30) is analyzed in Figure 5. In Figure 5, we explored whether the effect of divorce change is linked with the scale change through the violin plot..

All these applied divorce analyses prove to be very fruitful in the context of getting useful insights from the dataset and its related features.

The histogram chart is the plot of the dataset in Figures 6 and 7. A histogram is referred to as a data representation tool, which appears to be a bar chart that buckets a variation of outcomes along with the *x*-axis columns. The numerical value count or percent of value occurrences in the dataset for every column is represented on the *y*-axis.

We get the histogram of features 2_stranger (7), silence_instead_of_discussion (45), I'm_not_wrong (51), good_to_leave_home (44), I'm_not_guilty (50), humiliate (36), not_calm (37), negative_personality (33), and know_well (29) and get the total number of counts in the different scale values. The histogram is the plot of insult (35), common_goal (10), no_home_time (6), special_time (5), contact (4), begin_correct (3), ignore_diff (2), incompetence (54), always_never (32), and by counting the number of different scale values.

The histogram is the plot of the features friends_social (30), know_well (29), hopes_wishes (28), current_stress (27), anxieties (26), inner_world (25), fav_food (23), care_sack (22), and likes (21) showing the total number of counts on the *y*-axis and the 0 to 4 scale on the *x*-axis. The histogram chart is plotted on trust, role, marriage, love, and dreams columns and explored the number of counts on a different scale on the *y*-axis and *x*-axis, respectively.

From Figure 6, we have analyzed that the feature I'am_not_wrong (51) has higher rank values among all. This shows that this feature question has a major cause of divorce and that's why it has higher ranked scale values.

This applied divorce histogram analysis is based on the prominent questions present in the dataset and their scale ranks. These questions are analyzed to get their feature importance and to determine the relationship between divorce causes. These features are for model training and getting divorce prediction from it.

A correlation graph displays the correlations for various variables present in the dataset employed. The correlation matrix emphasizes the relationship between all the possible pairings of values in a dataset. It is a powerful tool for summarizing a large dataset in addition to visualizing and identifying trends in the provided data. We draw the correlation matrix on the dataset in Figure 8. The visualized features are based on the correlation values above or equal to 0.7. The feature that has low correlation values is not present in the feature display map. The correlation matrix shows that all features are highly related. All features are important to use for the training of our model.

### 3.3. Feature Engineering

The technique of changing the raw dataset into a prominent feature space that well describes the root problem of predictive techniques, resulting in improving the employed model accuracy results on the unseen dataset, is referred to as the feature engineering technique. The 54 features of the divorce questionnaire dataset are used as dependent features, and the target feature containing the label class is utilized in this research study. The top 10 absolute correlation features are examined in Figure 9. The fav_food (24), know_well (30), freedom_value (12), marriage (18), special_time (5), roles (19), harmony (11), happy (17), enjoy_travel (9), insult (36), humiliate (37), and trust (21) are the top correlated features.

### 3.4. Dataset Splitting

Dataset splitting appears as a requirement for removing bias from training data in machine learning systems. The dataset is split into two sets: the training dataset, which is used by the model to learn an efficient mapping of inputs to output, and the test set, which is utilized to effectively assess the proposed model's result performance. This division prevents the employed technique from overfitting [19]. The dataset splitting utilized in this research has a ratio of 80: 20. The 80% portion of the dataset is used to ensemble learning models, and the 20% portion of the dataset is utilized for testing and evaluating the ensemble model. The random state unit for splitting is 42.

## 4. Proposed Approaches

### 4.1. Passive Aggressive Classifier

The passive-aggressive categorization [20] is one of the accessible incremental learning methods because it uses a closed-form updating rule. In the sense that they do not require a learning rate, passive-aggressive algorithms are akin to perceptron models. They do, however, contain a regularization parameter. The classifier updates its weight vector for each misclassified training sample it gets in an attempt to fix it. The hyperparameters by tuning analysis of the passive-aggressive algorithm are examined in Table 2.

### 4.2. Support Vector Machine

The support vector machine (SVM) [21] is a supervised learning model that is utilized to solve regression and classification problems. It is largely employed in categorization-related difficulties. Every data item is visualized as a point in n-dimensional space, where *n* is the number of data features. The value of every data feature is the worth of a certain coordinate in the SVM model. Then, we achieve classification by establishing the hyper-plane that best distinguishes the two classes of the employed dataset. The SVM technique hyperparameters are analyzed in Table 3.

### 4.3. Neural Networks

A feedforward artificial neural network (ANN) that generates a set of outputs from a set of employed inputs is referred to as a multilayer perceptron (MLP) neural network [22]. An MLP is referred to by various layers of employed input nodes that are associated as a directed graph between the output and input layers. Backpropagation is utilized by MLP to train the employed neural network. An MLP is a neural network that joins many layers in a directed graph, which means that the data signal routed across the graph nodes is only a single direction. In addition to the input nodes, every node has an activation function of the nonlinear form.

Backpropagation [23] is a supervised machine learning technique utilized by an MLP. The MLP is a deep-learning-based approach since it uses various layers of neurons. The MLP is mostly utilized for supervised learning tasks, in addition to research into parallel distributed computing and computational neuroscience. Speech recognition, machine translation, and picture recognition are some of the applications of MLP. The hyperparameters analysis of MLP is examined in Table 4.

## 5. Ensemble Learning

The ensemble learning approach is examined and applied in this research. The architecture of the applied approach, the ensemble approach, is analyzed in Figure 10. The training dataset is used for training the three classification models utilized in this research. The SVM, linear model, and neural network model are trained and tested parallelly using the pipeline of ensemble learning. The ensemble learning architecture is based on the logic to train and test all model underlying models in parallel. Now, the testing results are used by the “hard” voting function to find the average accuracy of the model. We have applied hard voting because our classification data depends on class labels and the associated weights with every classifier. The higher accuracy score is our best prediction value.

## 6. Results and Evaluation

All performance evaluation metrics utilized in this research are examined in this section. The ensemble learning model accuracy score value, ROC accuracy score value, recall score value, precision score value, and F1 score values are the performance evaluation metrics employed in this research study. One parameter for assessing the classification models is accuracy. The accuracy score value is the percentage of the correct number of predictions made by our proposed model. The accuracy of our proposed technique is 100%. Formally, accuracy is represented by using the following mathematical equation:

(1) $$\begin{array}{c} \mathrm{accuracy}=\frac{\mathrm{number}\;\mathrm{of}\;\mathrm{correct}\;\mathrm{predictions}}{\mathrm{total}\;\mathrm{number}\;\mathrm{of}\;\mathrm{predictions}}. \end{array}$$

The ROC curve is referred to as the probability curve analysis that displays the true positive rate (TPR) outcome vs the false positive rate (FPR) outcome at numerous threshold settings, separating the signal data from the noise data. The area under the curve (AUC) is a measure of an employed learning classifier's ability to discriminate between classes and is utilized to summarize the ROC curve. The ROC AUC of our proposed technique is 97%. The mathematical equation expresses the ROC AUC score:

(2) $$\begin{array}{c} \text{ROC AUC}=\int_{0}^{1}\int_{-\infty }^{+\infty }{\text{ROC}}_{x}\left(t\right)dF_{\left(X|D=1\right)\left(x\right)dt}, \end{array}$$

(3) $$\begin{array}{c} \text{ROC AUC}=\int_{-\infty }^{+\infty }{\text{AUC}}_{x}dF_{\left(x|D=1\right)\left(x\right)}. \end{array}$$

Precision is referred to as the ratio of true positives rate (TPR) outcomes to all positive outcomes. The recall is a measure of how well our model identifies true positives. In our case, both have a 97% score. The mathematical equation that expressed the precision and recall:

(4) $$\begin{array}{c} \mathrm{precision}=\frac{\mathrm{true}\;\mathrm{positive}}{\mathrm{true}\;\mathrm{positive+false}\;\mathrm{positive}}, \end{array}$$

(5) $$\begin{array}{c} \mathrm{recall}=\frac{\mathrm{true}\;\mathrm{positive}}{\mathrm{true}\;\mathrm{positive+ false}\;\mathrm{negative}}. \end{array}$$

The F1 score value is measured by taking the weighted average value of recall and precision. As a result, this score value examines both the false positives rate (FPR) and the false negatives rate (FNR). The F1 score is periodically more valuable than the accuracy score value, exclusively if the dataset class distribution is not equal. In our situation, the F1 score is 97%. Mathematically, it is reparented as follows:

(6) $$\begin{array}{c} F1\;\mathrm{score}=2*\frac{\left(\mathrm{recall}\;*\;\mathrm{precision}\right)}{\left(\mathrm{recall}\;+\;\mathrm{precision}\right)}. \end{array}$$

The hyperparameter tuning results before and after are analyzed in Table 5. The k-fold cross validation comparative results are analyzed in Table 6. The applied learning techniques comparative analysis with the ensemble learning approach is demonstrated in Tables 7 and 8.

A confusion matrix (CM) analysis is referred to as a summary of the employed classification problem and the prediction outcomes as visualized in Figure 11. The number of right and wrong predictions is summarized with count values and divided by dataset category. The CM displays several methods in which the classification technique gets perplexed when making predictions. It is critical to assess the model's performance once it has been trained using some training data. When we developed a confusion matrix, we had several components:

- Positive (P): the projected outcome is positive (like the couple gets a divorce).
- Negative (N): the projected outcome is negative (like a couple does not get a divorce).
- True positive (TP): in this case, TP denotes the expected and actual values, which are both 1 (true).
- True negative (TN): TN denotes the projected value, while 0 denotes the actual value (false).
- False negative (FN): in this case, FN denotes that the predicted count value is 0 (N) while the actual count value is 1 (P). Both values in this case do not correspond. As a result, it is an FN.

## 7. Conclusion

The prediction of divorce by using machine learning and ensemble learning techniques is the core motive of this research study. The findings of our study are based on key indicators for divorce and the factors that are most significant when predicting divorce. The support vector machine (SVM), passive aggressive classifier, and neural network (MLP) are applied to predict divorce. The cross-validation and performance evaluation techniques are manipulated to evaluate the proposed models. Our EL proposed technique achieved the highest accuracy of 100%. In the context of limitations and future directions, we will try to enhance the questionnaire dataset by adding more questions to get more clarified results and also apply the data augmentation techniques. To reduce overfitting, we will explore different deep learning models.

## Figures and Tables

**Figure 1:** The methodology diagram of the proposed research system.

**Figure 2:** The divorce dataset balancing analysis by the target class.

**Figure 3:** Divorce analysis by I'm_not_wrong, enjoy_holiday, love, and common_goals features. (a) The violin graph analysis of I'm_not_wrong feature among Divorced and not Divorced category, (b) The violin graph analysis of enjoy_holiday feature among Divorced and not Divorced category, (c) The violin graph analysis of love feature among Divorced and not Divorced category, and (d) The violin graph analysis of common_goals feature among Divorced and not Divorced category.

**Figure 4:** Divorce analysis by happy, always_never, trust, and you're_inadequate features. (a) The violin graph analysis of happy feature among Divorced and not Divorced category, (b) The violin graph analysis of always_never feature among Divorced and not Divorced category, (c) The violin graph analysis of trust feature among Divorced and not Divorced category, and (d) The violin graph analysis of you're_inadequate feature among Divorced and not Divorced category.

**Figure 5:** The divorce analysis by argue_then_leave, humiliates, and friends_social features. (a) The violin graph analysis of argue_then_leave feature among Divorced and not Divorced category, (b) The violin graph analysis of humiliates feature among Divorced and not Divorced category, (c) The violin graph analysis of friends_social feature among Divorced and not Divorced category.

**Figure 6:** The divorce histogram analysis of 15 prominent questions scale ranks analysis. (a) The ranked scale analysis being the lowest and highest for feature Ignore_diff, (b) The ranked scale analysis being the lowest and highest for feature incompetence, (c) The ranked scale analysis being the lowest and highest for feature Always_never, (d) The ranked scale analysis being the lowest and highest for feature friends_social, (e) The ranked scale analysis being the lowest and highest for feature hopes_wishes, (f) The ranked scale analysis being the lowest and highest for feature current_stress, (g) The ranked scale analysis being the lowest and highest for feature anxieties, (h) The ranked scale analysis being the lowest and highest for feature inner_world, (i) The ranked scale analysis being the lowest and highest for feature fav_food, (j) The ranked scale analysis being the lowest and highest for feature care_sick, (k) The ranked scale analysis being the lowest and highest for feature likes, (l) The ranked scale analysis being the lowest and highest for feature trust, (m) The ranked scale analysis being the lowest and highest for feature roles, (n) The ranked scale analysis being the lowest and highest for feature marriage and (o) The ranked scale analysis being the lowest and highest for feature love.

**Figure 7:** The divorce histogram analysis of other 15 prominent questions scale ranks analysis. (a) The ranked scale analysis being the lowest and highest for feature dreams, (b) The ranked scale analysis being the lowest and highest for feature incompetence, (c) The ranked scale analysis being the lowest and highest for feature Always_never, (d) The ranked scale analysis being the lowest and highest for feature friends_social, (e) The ranked scale analysis being the lowest and highest for feature hopes_wishes, (f) The ranked scale analysis being the lowest and highest for feature current_stress, (g) The ranked scale analysis being the lowest and highest for feature anxieties, (h) The ranked scale analysis being the lowest and highest for feature inner_world, (i) The ranked scale analysis being the lowest and highest for feature fav_food, (j) The ranked scale analysis being the lowest and highest for feature care_sick, (k) The ranked scale analysis being the lowest and highest for feature likes, (l) The ranked scale analysis being the lowest and highest for feature trust, (m) The ranked scale analysis being the lowest and highest for feature roles, (n) The ranked scale analysis being the lowest and highest for feature marriage and (o) The ranked scale analysis being the lowest and highest for feature love.

**Figure 8:** Dataset correlation analysis.

**Figure 9:** The top 10 absolute correlation feature analyses.

**Figure 10:** The proposed ensemble learning architecture analysis.

**Figure 11:** The proposed ensemble learning approach confusion matrix.

**Table 1:** The dataset attribute details.

Question no.	Question by the specialist
1	If one of us apologizes when our discussion deteriorates, the discussion ends.
2	I know we can ignore our differences, even if things get hard sometimes.
3	When we need it, we can take our discussions with my spouse from the beginning and correct them.
4	When I discuss this with my spouse, contacting him will eventually work.
5	The time I spent with my wife is special for us.
6	We don't have time at home as partners.
7	We are like two strangers who share the same environment at home rather than family.
8	I enjoy our holidays with my wife.
9	I enjoy traveling with my wife.
10	Most of our goals are common to my spouse.
11	I think that one day in the future when I look back, I see that my spouse and I have been in harmony with each other.
12	My spouse and I have similar values in terms of personal freedom.
13	My spouse and I have a similar sense of entertainment.
14	Most of our goals for people (children, friends, etc.,) are the same.
15	Our dreams with my spouse are similar and harmonious.
16	We're compatible with my spouse about what love should be.
17	We share the same views about being happy in our life with my spouse.
18	My spouse and I have similar ideas about how marriage should be.
19	My spouse and I have similar ideas about how roles should be in marriage.
20	My spouse and I have similar values in trust.
21	I know exactly what my wife likes.
22	I know how my spouse wants to be taken care of when she/he is sick.
23	I know my spouse's favorite food.
24	I can tell you what kind of stress my spouse is facing in her/his life.
25	I know my spouse's inner world.
26	I know my spouse's basic anxiety.
27	I know what my spouse's current sources of stress are.
28	I know my spouse's hopes and wishes.
29	I know my spouse very well.
30	I know my spouse's friends and their social relationships.
31	I feel aggressive when I argue with my spouse.
32	When discussing with my spouse, I usually use expressions such as “you always” or “you never.”
33	I can use negative statements about my spouse's personality during our discussions.
34	I can use offensive expressions during our discussion.
35	I can insult my spouse during our discussion.
36	It can be humiliating when we have discussions.
37	My discussion with my spouse is not calm.
38	I hate my spouse's way of opening a subject.
39	Our discussions often occur suddenly.
40	We're just starting a discussion before I know what's going on.
41	When I talk to my spouse about something, my calm suddenly breaks.
42	When I argue with my spouse, I only go out and I do not say a word.
43	I mostly stay silent to calm the environment a little.
44	Sometimes I think it's good for me to leave home for a while.
45	I'd rather stay silent than discuss it with my spouse.
46	Even if I'm right in the discussion, I stay silent to hurt my spouse.
47	When I discuss this with my spouse, I stay silent because I am afraid of not being able to control my anger.
48	I feel right in our discussions.
49	I have nothing to do with what I have been accused of.
50	I'm not the one who's guilty of what I am accused of.
51	I'm not the one who's wrong about problems at home.
52	I wouldn't hesitate to tell my spouse about her/his inadequacy.
53	When I discuss, I remind my spouse of her/his inadequacy.
54	I'm not afraid to tell my spouse about her/his incompetence.

**Table 2:** The applied model hyperparameters by tuning.

Proposed technique	Hyperparameters		
	Max iterations	Verbose	Random state
Passive aggressive classifier (PAC)	300	0	50

**Table 3:** The applied model hyperparameters by tuning.

Proposed technique	Hyperparameters		
	Max iterations	Kernel	Random state
Support vector machine (SVM)	300	Linear	10

**Table 4:** The applied model hyperparameters by tuning.

Proposed technique	Hyperparameters					
	Hidden layers	Activation	Random state	Verbose	Max iterations	Solver
Neural networks (MLP)	200	Logistic	50	0	200	Adam

**Table 5:** The comparison analysis of selected methods before and after hyperparameter tuning.

Proposed technique	Before hyperparameter tuning		After hyperparameter tuning	
	Accuracy score	Training time (seconds)	Accuracy score	Training time (seconds)
Support vector machine (SVM)	97	0.004660367965698242	100	0.0017824172973632812
Passive aggressive classifier (PAC)	97	0.0012810230255126953	97	0.002166748046875
Neural network (MLP)	97	0.9576735496520996	100	0.4841580390930176

**Table 6:** The *k*-fold cross-validation results of applied machine learning approaches.

Sr. no.	Proposed technique	Accuracy score %
1	Support vector machine (SVM)	98
2	Passive aggressive classifier (PAC)	98
3	Neural network (MLP)	98

**Table 7:** The comparative analysis of the proposed ensemble techniques.

Proposed technique	Comparative analysis metrics		
	Accuracy %	Log loss	Training time (seconds)
Support vector machine (SVM)	100	9.992007221626415*e* − 16	0.0017824172973632812
Passive aggressive classifier (PAC)	97	1.0158463645561975	0.002166748046875s
Neural network (MLP)	100	9.992007221626415*e* − 16	0.4841580390930176
Ensemble learning (EL)	100	9.992007221626415*e* − 16	1.0685508251190186

**Table 8:** The ensemble learning performance evaluation results.

Proposed technique	Performance evaluation metrics					
	Accuracy %	ROC accuracy %	Precision accuracy %	Recall accuracy %	F1 score %	Log loss
Ensemble learning (EL)	100	97	97	97	97	9.992007221626415*e* − 16

## Data Availability

The supporting data for the findings of this study are available from the corresponding author on reasonable request.
